# m6A-Mediated Tumor Invasion and Methylation Modification in Breast Cancer Microenvironment

**DOI:** 10.1155/2021/9987376

**Published:** 2021-10-27

**Authors:** Fei Liu, Xiaopeng Yu, Guijin He

**Affiliations:** Shengjing Hospital of China Medical University, Shenyang 110013, China

## Abstract

**Background:**

We analyzed the n6-methyladenosine (m6A) modification patterns of immune cells infiltrating the tumor microenvironment of breast cancer (BC) to provide a new perspective for the early diagnosis and treatment of BC.

**Methods:**

Based on 23 m6A regulatory factors, we identified m6A-related gene characteristics and m6A modification patterns in BC through unsupervised cluster analysis. To examine the differences in biological processes among various m6A modification modes, we performed genomic variation analysis. We then quantified the relative infiltration levels of different immune cell subpopulations in the tumor microenvironment of BC using the CIBERSORT algorithm and single-sample gene set enrichment analysis. Univariate Cox analysis was used to screen for m6A characteristic genes related to prognosis. Finally, we evaluated the m6A modification pattern of patients with a single BC by constructing the m6Ascore based on principal component analysis.

**Results:**

We identified three different m6A modification patterns in 2128 BC samples. A higher abundance of the immune infiltration of the m6Acluster C was indicated by the results of CIBERSORT and the single-sample gene set enrichment analysis. Based on the m6A characteristic genes obtained through screening, the m6Ascore was determined. The BC patients were segregated into m6Ascore groups of low and high categories, which revealed significant survival benefits among patients with low m6Ascores. Additionally, the high-m6Ascore group had a higher mutation frequency and was associated with low PD-L1 expression, and the m6Ascore and tumor mutation burden showed a positive correlation. In addition, treatment effects were better in patients in the high-m6Ascore group.

**Conclusions:**

In case of a single patient with BC, the immune cell infiltration characteristics of the tumor microenvironment and the m6A methylation modification pattern could be evaluated using the m6Ascore. Our results provide a foundation for improving personalized immunotherapy of BC.

## 1. Introduction

As a common malignant tumor amongst women, breast cancer (BC) happens to be the fifth leading reason for cancer-related mortalities across the world. Of all cancer cases, 11.7% or approximately 2.3 million new cases of BC were recorded in 2020, and the incidence of female BC is increasing each year [1, 2]. Diagnostic and treatment advancements have recently led to substantial reductions in the mortality rate of BC [3]. However, many patients with BC have a poor prognosis. Studies of the tumor microenvironment (TME) have clarified the roles of key immune cell subgroups in the occurrence and development of cancer [4–6]. Harao et al. found a significant link between the density of CD8+ T cells and immune escape of BC, as well as the infiltration of CD4+ T cells and CD8+ T cells with BC prognosis [7]. In addition, specific immune checkpoint inhibitors such as CTLA-4, PD-1, and PD-L1 have dramatically changed the current status of cancer treatment and are beneficial for the overall survival (OS) of a variety of patients with cancer [8, 9]. CTLA-4-, PD-1-, and PD-L1-specific antagonists have also made progress in clinical trials of BC [10, 11]. For developing new immunotherapeutic strategies and predicting the response to the existing immune checkpoint inhibitors, it is crucial to assess the immune infiltration based on the characteristics of the TME [12–14]. Therefore, by comprehensively analyzing the complexity and heterogeneity of the TME, potential biomarkers can be identified to help guide and predict the response to immunotherapy [13, 15].

Among more than 100 RNA modifications, the most common is n6-methyladenosine (m6A) [16]. In global cellular RNA, m6A occurs on 0.2–0.4% of all adenosine and approximately 50% of all methylated ribonucleotides [17]. Modification of m6a regulates addition, removal, and recognition through methyltransferase “writers,” demethylase “erasers,” and binding protein “readers,” respectively [18–21]. Previous studies showed that m6 methylation can regulate mRNA splicing, expression, nuclear export, and translation and has an important role in the development of tumors [22–25]. Many previous studies demonstrated that m6A methylation can regulate mRNA splicing, expression, decay, and translation and plays an important role in various cellular pathways and biological processes [26, 27]. For early diagnosis and treatment of cancer, the m6A methylation provides a new perspective.

The action mechanism between m6A modification and the TME-infiltrating immune cells could not be explained as revealed also from the earlier studies on the mechanism of the RNA degradation. YTHDF1 in dendritic cells can recognize and bind m6A-modified mRNA encoding lysosomal cathepsin, promote cathepsin translation, and inhibit the cross-initiation of dendritic cells [28]. Li et al. found that the absence of the m6A demethylase ALKBH5 enhanced the sensitivity of tumors to cancer immunotherapy and improved the efficacy of immunotherapy [29]. ALKBH5 can affect the lactic acid content of the tumor microenvironment, tumor-infiltrating Tregs, and myeloid-derived suppressor cells by regulating the expression and splicing of target genes. Yang et al. suggested that increased FTO expression can promote the growth of melanoma by reducing m6A methylation in PD-1, CXCR4, and SOX10 and preventing their RNA from YTHDF2-mediated decay [30]. Knockout of FTO in melanoma cells increased the sensitivity of tumor cells to interferon gamma and enhanced the response of mice to anti-PD-1 antibodies. However, previous studies focused on only a few m6A regulatory factors and the antitumor effects of these regulatory factors are achieved in a highly coordinated manner by many tumor suppressors. Additionally, m6A regulatory factors can be comprehensively evaluated if transcriptomic and genomic data are accumulated, such as through high-throughput sequencing analysis. Therefore, identifying and analyzing the characteristics of TME cell infiltration mediated by multiple m6A regulatory factors are beneficial for promoting immunotherapy development [31, 32].

In this study, we used the Gene Expression Omnibus (GEO) and The Cancer Genome Atlas (TCGA) databases to download the clinical information and transcriptome data of 2128 BC samples. The association between the TME cell infiltration and the m6A modification patterns was analyzed comprehensively. Three distinct patterns of m6A modification were detected, and hence, to measure the patterns of the m6A modification of BC, a scoring scheme was developed. Our results indicate that m6A modification is important for improving current BC treatments.

## 2. Materials and Methods

### 2.1. Collection of BC Data

Using the GEO (http://www.ncbi.nlm.nih.gov/geo/) and TCGA (https://tcga-data.nci.nih.gov/tcga/) databases, we collected clinical information and transcriptome data on BC samples. We included seven datasets, specifically GSE48390.txt, GSE58812.txt, GSE88770.txt, GSE131769, GSE42568, GSE20685, and TCGA-BC. Downloading of the genomic mutation data of the patients with BC was done from the database of the TCGA. For the TCGA-BC dataset, we used the *R* package TCGAbiolinks to convert the fragments per kilobase of transcript per million mapped reads value into a transcript with a million per thousand base value [33]. The *R* package “SVR” was employed to manage batch effects among various datasets [34]. The copy number variation (CNV) map of the 23 m6A regulators on the human chromosome was generated using the *R* package “RCircos.”

### 2.2. Cluster Analysis of 23 m6A Modulators

We collected 23 m6A regulatory genes, including eight writers (METTL3, METL14, METL16, WTAP, VIRMA, ZC3H13, RBM15, and RBM15B), 13 readers (YTHDC1, YTHDC2, YTHDF1, YTHDF2, YTHDF3, HNRNPC, FMR1, LRPPRC, HNRNPA2B1, IGFBP1, IGFBP2, IGFBP3, and RBMX), and two erasers (FTO and ALKBH5).

To determine the various patterns of the m6A modification, an unsupervised cluster analysis was conducted, based on the 23 m6A regulatory genes. The optimal number of clusters was selected according to the coefficients of contour, dispersion, and symbiosis. The *R* package ConsensusClusterPlus was utilized to perform the cluster analysis.

### 2.3. Functional Annotation and Gene Set Variation Analysis

Using the *R* package “GSVA,” gene set variation analysis (GSVA) enrichment analysis was performed to examine the differences in biological processes among the various m6A modification modes. For GSVA, we downloaded the gene set of “h.all.v7.4.symbols.gmt” from the MSigDB database [35]. Using the *R* package “clusterProfiler,” the functional annotation was conducted. A false discovery rate of <0.05 was set as the cutoff value.

### 2.4. Analysis of Immune Cell Infiltration between Different m6A Modification Modes

The relative abundance of each immune cell type infiltrating the TME of BC was determined by conducting a single-sample gene set enrichment analysis. We evaluated activated CD8 T cells, activated dendritic cells, macrophages, natural killer T cells, and regulatory T cells. Using the enrichment score obtained from the single-sample gene set enrichment analysis, the relative abundance of each immune cell type was specified.

### 2.5. Analysis of Differentially Expressed Genes between Different Types of m6A

Patients with BC were clustered into three groups based on different m6A modification patterns. To identify the differentially expressed genes (DEGs) between the modes of the three m6A modifications, the *R* package “limma” was used [36]. A *P* < 0.001 was considered to indicate a DEG.

### 2.6. Construction of m6A Gene Signature

First, we used univariate Cox for gene prognosis analysis based on the overlapping DEGs between different m6Aclusters and selected genes, with significant effects on prognosis for subsequent analysis, with *P* < 0.05 as the cutoff value. Segregating the patients into three groups for subsequent analysis, to analyze the prognostic-related genes, an unsupervised clustering method was applied. Finally, the gene expression profiles for principal component analysis were consolidated, and principal components 1 and 2 were extracted as feature scores. This method primarily concentrates on the score of the set with the most significantly correlated or inversely correlated gene block in the set. Simultaneously, it weighs the contribution of untracked genes to other set members. We constructed the m6A gene signature using a previously described formula [37, 38], m6Ascore = ∑(PC1i + PC2i), where *i* is the expression of genes related to the m6A phenotype.

### 2.7. Statistical Analysis

R-3.4.2 was used for statistical analysis. To determine the differences between the multiple groups, the one-way analysis of variance and the Kruskal–Wallis test were conducted [39]. For segregating the samples into low- and high-m6Ascore groups, the “surv-cutpoint” function was applied. The Kaplan–Meier method was used to draw the survival curve for prognostic analysis. The waterfall function in MAFtools package was used to evaluate the mutation status of both groups of patients, specifically those with low- and high-m6Ascore subtypes. The result with *P* value <0.05 was considered to be statistically significant.

## 3. Results

### 3.1. m6A Regulators in BC and Their Genetic Variation Landscape

We studied the role of 23 m6A regulatory genes in BC, including eight writers (METTL3, METL14, METL16, WTAP, VIRMA, ZC3H13, RBM15, and RBM15B), 13 readers (YTHDC1, YTHDC2, YTHDF1, YTHDF2, YTHDF3, HNRNPC, FMR1, LRPPRC, HNRNPA2B1, IGFBP1, IGFBP2, IGFBP3, and RBMX), and two erasers (FTO and ALKBH5). First, we determined the incidence of CNV and somatic mutations in 23 m6A regulatory factors in BC.  Figure 1(a) shows that 57 of 986 samples had mutations in the m6A regulatory factor, with a frequency of 5.78%. A mutation frequency of 1% was observed in YTHDF3, WTAP, HNRNPA2B1, FMR1, YTHDF1, RBM15, LRPPRC, and ZC3H13. Five writers (METTL3, METL14, METL16, VIRMA, and RBM15B), eight readers (YTHDC1, YTHDC2, YTHDF2, HNRNPC, IGFBP1, IGFBP2, IGFBP3, and RBMX), and two erasers (FTO and ALKBH5) were not mutated. Further analysis of the 23 m6A regulatory factors in BC revealed that CNV mutations in 23 m6A regulatory factors were common. VIRMA, YTHDF1, YTHDF3, HNRNPC, METL3, YTHDC1, FTO, FMR1, and RBMX showed extensive CNV amplification. In contrast, WTAP, RBM15, ZC3H13, YTHDF2, and RBM15B contained common CNV deletions (Figure 1(b)).  Figure 1(c) shows the changes in the positions of the CNVs of the 23 m6A regulatory factors in human chromosomes. Around 23 m6A regulators completely distinguished the BC tumor samples from the normal samples by performing the principal component analysis of the BC samples (Figure 1(d)). Additionally, in patients with BC, by exploring the mRNA expression levels of these factors between the tumor and the normal samples, we could determine if the expression of the m6A regulatory factors was impacted by the genetic variations above. The results indicate that changes in CNV lead to changes in m6A regulatory factors. The expression of METTL14, METTL16, WTAP, ZC3H13, YTHDC1, IGFBP1, IGFBP3, and FTO in normal tissues was higher than that in tumor tissues. In contrast, the expression of VIRMA, RBM15, YTHDF1, YTHDF2, HNRNPC, FMR1, LRPPRC, HNRNPA2B1, and IGFBP2 in tumor tissues was higher than that in normal tissues (Figure 1(e)). These results show that the genetic variation and expression of m6A regulatory factors significantly differed between tumor and normal samples and may be vital for BC development and occurrence.

### 3.2. Pattern of m6A Modification in BC Was Mediated by 23 Regulatory Factors

We included seven datasets with clinical information (TCGA-BC, GSE48390.txt, GSE58812.txt, GSE88770.txt, GSE20685, GSE42568, and GSE131769) for subsequent analysis.  Figure 2(a) shows the m6A regulatory factor network, which revealed interactions between 20 m6A regulatory factors and the prognostic significance of the regulatory factors in patients with BC. A significant correlation was found among the m6A regulators in the same category, as well as in erasers, readers, and writers. In the formation of distinct m6A modification patterns, the link between erasers, readers, and writers may be vital and impact the development and occurrence of BC. We next performed unsupervised cluster analysis based on the expression of m6A regulatory factors to classify samples with different m6A modification patterns and finally determined three different modification patterns: m6Acluster A (494 cases), m6Acluster B (940 cases), and m6Acluster C (694 cases) (Figures 2(b)–2(d)).

### 3.3. Immune Landscape Features in Different m6A Modification Modes

The GSVA for enrichment was performed to investigate the biological behaviors of the three different m6A modification modes (Figures 3(a)–3(c)). The results of GSVA showed that m6Acluster A showed a higher association with protein secretion, mitotic spindle, and G2M checkpoint. m6Acluster B showed a higher association with myogenesis, KRAS signaling, and estrogen response late. m6Acluster C showed a higher association with allograft rejection, complement, IL-6 JAK STAT3 signaling, inflammatory reaction, and interferon-*γ* reaction. In addition, we used the deconvolution algorithm CIBERSORT to further evaluate the immune infiltration characteristics of the three m6A modification patterns. The results showed that m6Acluster C had better stromal scores, immune scores, and ESTIMATE scores (Figure 3(d)). We also performed single-sample gene set enrichment analysis to determine the TME immune cell infiltration of BC, with the results showing that immune cell infiltration in m6Acluster C was more abundant, including natural killer cells, macrophages, mast cells, and plasmacytoid dendritic cells (Figure 3(e)).

### 3.4. m6A Phenotype-Related DEGs in BC

Three different m6A modification patterns showed distinct differences in the m6A transcription profile (Figure 4(a)). Although unsupervised cluster analysis based on the expression of m6A regulatory factors divided patients with BC into three different m6A modification patterns, the underlying genetic changes and mechanism of action were unclear. Therefore, we applied the empirical Bayes method to screen DEGs that overlapped between the three m6A modification patterns, revealing 2124 DEGs (Figure 4(b)). We also performed gene function enrichment analysis of these DEGs. Gene ontology enrichment analysis showed that biological processes such as cilium organization, transcription corepressor activity, and ubiquitin protein ligase activity were significantly upregulated (Figure 4(c)). Kyoto Encyclopedia of Genes and Genomes enrichment analysis showed that biological processes such as ubiquitin-mediated proteolysis, *Salmonella* infection, endocytosis, and AMPK signaling pathway were significantly upregulated (Figure 4(d)). Furthermore, we performed unsupervised cluster analysis based on the DEGs to verify this adjustment mechanism. To screen the DEGs related to prognosis, the univariate Cox analysis was conducted which revealed 668 DEGs with *P* < 0.05. Next, we performed unsupervised cluster analysis based on the 668 genes and divided the patients into three different genomic subtypes (gene clusters I–III) (Figures 5(a)–5(c)). The clustering results supported that there were three different m6A methylation modification patterns in BC.  Figure 5(d) shows evident cluster separation between the three gene clusters.  Figure 5(e) shows the different clinicopathological characteristics of these subgroups. Subsequent survival analysis revealed significant prognostic differences between the three different clusters and that gene cluster II was associated with better survival results (Figure 5(f)). In addition, between the three different gene clusters, the estimated results of the m6A methylation modification pattern were found to be consistent with the significant differences in the expression of the m6A regulatory factors (Figure 5(g)). We also conducted single-sample gene set enrichment analysis, which showed that immune cells in gene cluster III were more permeable, including B cells, CD4 T cells, CD8 T cells, dendritic cells, natural killer cells, and MDSCna (Figure 5(h)).

### 3.5. m6A Gene Signature, Function Annotation, and Clinical Significance

The findings described above were based on patient populations and thus could not accurately predict the m6A modification pattern in a specific patient sample. Therefore, to quantify the m6A pattern of a single patient with BC, a scoring system (m6Ascore) was developed. Alluvial plots were used to show the changes in the characteristics of patients with BC (Figure 6(a)).  Figure 6(b) shows the correlation between the m6Ascore and immune cells. The results showed that m6Ascore was positively correlated with natural killer cells, MDSCna, macrophagena, and monocytena. The Kruskal–Wallis test showed that the m6Ascore and m6Acluster significantly differed. The m6Ascore of m6Acluster B was significantly higher than that of m6Acluster A (Figure 6(c)). In addition, compared with other m6A gene clusters, gene cluster III showed the highest m6Ascore, whereas gene cluster II had the lowest m6Ascore (Figure 6(d)). These results showed that the m6Ascore can be used to evaluate the m6A modification pattern of a single BC and TME immune cell infiltration characteristics of the tumor. We also analyzed the value of m6Ascore for predicting patient survival outcomes. The survival results showed that patients with low m6Ascore showed significant survival benefits (Figure 6(e)).

There is increasing evidence of a correlation between somatic mutations in tumor genomes and the immunotherapy response. Analysis of the distribution pattern of tumor mutation burden (TMB) in different m6Ascore groups showed that the mutation frequency of the high-m6Ascore group was higher than that of the low-m6Ascore group (Figure 6(f)).  Figure 6(g) shows that the m6Ascore and TMB were positively correlated (*R* = 0.26, *P*=8*e* − 16). Compared to the patients of the high-TMB group, the low-TMB group patients indicated better survival results (Figure 6(h)). In addition, regardless of whether the m6Ascore was high or low, patients in the low-TMB group consistently showed a significant survival advantage (Figure 6(i)). Variations in the distribution of somatic mutations between the high- and low-m6Ascore groups were evaluated using the MAFtools package. The former group illustrated a broader TMB compared to the latter group in the results (Figures 6(j) and 6(k)). These results improve the understanding of the impact of m6Ascore classification on genomic variation and reveal a potential interaction of individual somatic mutations and m6A modifications.

### 3.6. Predictive Value of m6Ascore on the Effect of Immunotherapy

Immunosuppressive agents can improve cancer treatment. Both the Tumor Immune Dysfunction and Exclusion (TIDE) and immunophenoscore, which are recently discovered predictors, have been broadly applied to assess immune responses. We analyzed the expression of TIDE in the low- and high-m6Ascore groups. Compared to the high-m6Ascore group, the TIDE of the low-m6Ascore group was found to be lower, as per the results (*P*=0.042) (Figure 7(a)). In the CTLA-4 and PD-1 groups, patients in the high-m6Ascore group showed better treatment effects (CTLA-4: *P* = 1.2e−12; PD-1: *P* = 5.4e−08) (Figures 7(b) and 7(c)). In the CTLA-4 and PD-1 combined treatment group, patients in the high-m6Ascore group still exhibited better treatment effects (*P* = 1.5e−09) (Figure 7(d)). Additionally, low PD-L1 expression was observed among patients with high m6Ascores, indicating that these patients will respond to anti-PD-1/L1 immunotherapy (Figure 7(e)). In the mediating immune responses, the significant role played by the m6A modification modes of BC was supported by these results.

## 4. Discussion

Previous studies showed that the interaction between m6A modification and m6A regulatory factors is important in various cancer functions, including cancer stem cell formation, epithelial-mesenchymal transition, cancer metabolism, and signal transduction [40–43]. As most previous studies focused on a single m6A regulatory factor, the characteristics of TME immune infiltration mediated by multiple m6A regulatory factors are unclear. Thus, identifying the function of m6A modification patterns in TME immune cell infiltration is fundamental for improving the understanding of the interaction between m6A RNA and antitumor immune responses and facilitating the advancement of personalized treatments for patients with BC.

The genetic variation in the m6A regulatory factor in BC shows that eight regulatory factors (YTHDF3, WTAP, HNRNPA2B1, FMR1, YTHDF1, RBM15, LRPPRC, and ZC3H13) have mutations. In RNA stability, editing, translating, splicing, processing, and regulation, the Pentagram Peptide Repeat (PPR) family was found to play a significant role. LRPPRC is a multifunctional protein in the PPR family [44]. The increases in the various cell lines and the cancer tissues of the LRPPRC expression were illustrated by the earlier studies too [45–49]. MAP1S of the microtubule-associated protein family can link mitochondria and microtubules for transport and affect the biogenesis and degradation of autophagosomes, thereby increasing autophagy and inhibiting tumorigenesis. The combination of high expression of LRPPRC and low expression of MAP1S can inhibit autophagy and promote tumor development [50]. ZC3H13 is a classic CCCH zinc finger protein. Previous studies have demonstrated that ZC3H13 may be a tumor suppressor protein and has somatic mutations in colon cancer [51]. YTHDF1 is an important regulator of m6A methylation and can promote the translation of the key Wnt receptor frizzled7 in an m6A-dependent manner. In addition, mutations in YTHDF1 can enhance the expression of frizzled7, leading to excessive activation of the Wnt/*β*-catenin pathway and promoting gastric cancer [52]. However, our understanding of the role of these m6A regulatory factor mutations in BC is limited, and more experiments are needed.

Based on 23 m6A regulatory factors, three distinct m6A modification patterns were identified. The Hallmark gene set in the Molecular Characteristics Database (MSigDB) summarizes and represents a specific well-defined biological state or process. We performed GSVA analysis based on h.all.v7.4.symbols.gmt, and the results showed that m6Acluster A was more related to cell pathway and proliferation. m6Acluster B was more related to cell development and signaling. In m6Acluster C, immune-related pathways were more active. The IL-6 JAK STAT3 pathway has been shown to have an important effect on the development of various human tumors [53]. IL-6, as the main medium of inflammation, is highly expressed in tumor microenvironment. STAT3 is a member of the STAT protein family and is significantly associated with promoting tumor development and immunosuppression [54, 55]. JAK/STAT3 signaling pathways play an important role in mediated IL-6 inhibition of tumor cell proliferation, invasion, and metastasis and antitumor immunity. Previous cumulative studies have found that increased expression of IL-6 stimulates overactivation of JAK/STAT3 signals and leads to poor prognosis in cancer patients [56–58]. Previous studies showed that the expression levels of tumor-infiltrating CD4+ T cells, CD8+ T cells, macrophages M1, and natural killer cells may be related to the immune response [12, 59, 60]. Our results confirmed that the m6Acluster C pattern is associated with increased levels of tumor-infiltrating immune cells. A highly significant correlation indicated the potential value for supporting immunotherapy. Previous studies showed that STAT inhibitors can inhibit STAT3 protein expression in lymphoma and have early clinical activity. In addition, patients with lymphoma show decreased tumor cells and myeloid-derived suppressor cells and increased CD8+ T cells [61]. Therefore, patients with BC in m6Acluster C mode may benefit from treatment with STAT blockers.

Gene function enrichment analysis showed that the potential biological pathways of DEGs between the three different m6A clusters were significantly related. This indicates that these DEGs are characteristic genes related to the m6A phenotype. Prognostic-related m6A signature genes were screened and used to identify three genomic subtypes, which are also related to different TME immune landscapes in BC. In addition, for quantifying the m6A modification pattern of a single BC intended to improve the personalized treatment, a scoring system (m6Ascore) was developed. Patients with a low m6Ascore exhibit obvious survival advantages. In addition, our results also showed that the m6Ascore was significantly correlated with predictors of the immune response such as PD-L1, immunophenoscore, and TIDE, indicating that modification of m6A impacts the therapeutic effect of immunotherapy and is conducive for improving personalized treatment of BC. CTLA-4-, PD-1-, and PD-L1-specific immune checkpoint antagonists have completely improved the current status of cancer treatment. The FDA has approved several drugs for the treatment of a variety of cancers, but no immune checkpoint antagonist drug has been approved for the treatment of breast cancer. Even so, there are some CTLA-4 antagonists and PD-1/PD-L1 antagonist drugs, such as ipilimumab, avelumab, and pembrolizumab, which are currently entering BC clinical trials. In certain patients with metastatic BC, the PD-1/PD-L1 antagonist drugs were found to induce a durable clinical response, as research has revealed [10]. Therefore, our results need to be verified in more immunotherapy treatment cohorts in the future.

Exploring mutation driver genes in tumors will enable the development of cancer diagnosis and treatment approaches. We also analyzed the correlation between the m6Ascore and tumor mutation burden. In the high-m6Ascore group, the mutation frequencies of TP53, PIK3CA, and TTN were highest. In the low-m6Ascore group, the mutation frequencies of PIK3CA, TP53, and TTN were highest. Previous studies showed that PIK3CA is commonly mutated in BC [62] and that this mutation is highly heterogeneous in BC. In addition, in BC, the proportion of HR+/HER2-subtypes was highest, followed by the HER2+ and triple-negative BC subtypes [63]. Mosele et al. showed that patients with the PIK3CA mutant HR+/HER2-subtype have a poor prognosis and are resistant to chemotherapy. In contrast, patients with the PIK3CA mutant triple-negative BC subtype have a clear survival advantage [64]. TP53 (P53) is a tumor suppressor gene that is frequently mutated in various cancers [65]. Mutations in P53 in cancer can affect the activity and recruitment of bone marrow and T cells, leading to immune evasion, thereby promoting the occurrence and development of tumors. P53 can also affect tumor occurrence and development by acting on immune cells [66]. The mechanism of action underlying m6A modification and these tumor mutant genes requires further analysis.

Our study had some limitations. First, we did not evaluate a large number of clinicopathological features. Second, larger cohorts of patients with BC being treated with immunotherapy should be examined to verify our results.

## 5. Conclusion

In summary, the m6Ascore can be used to evaluate the m6A modification pattern and TME immune cell infiltration characteristics of a single patient with BC and is useful for predicting the survival outcome of patients with BC. Moreover, the clinical response to immunotherapy can be predicted using the m6Ascore. Our results provide insight for improving personalized cancer immunotherapy.

## Figures and Tables

**Figure 1:** Genetic mutation landscape of m6A regulatory factors in breast cancer. (a) The mutation frequency of 23 m6A regulatory factors in 986 patients with breast cancer in the TCGA-BC cohort was 5.78%. Each column represents a single patient. The bar graph above shows the tumor mutation burden, and the numbers on the right indicate the mutation frequency of each regulator. (b) Copy number variation mutation frequency of m6A regulator (blue dot, delete frequency; red dot, amplify frequency). (c) Position of copy number variation change of m6A regulatory factor on human chromosome. (d) Principal component analysis was performed on m6A regulators in the TCGA-BC cohort to distinguish tumors from normal samples. Tumor and normal samples are marked in blue and red, respectively. (e) Difference in the expression level of m6A regulatory factors between normal and tumor samples. Blue and red represent normal and tumor samples, respectively (^*∗*^*P* < 0.05, ^*∗∗*^*P* < 0.01, and ^*∗∗∗*^*P* < 0.001).

**Figure 2:** Pattern of m6A methylation modification in breast cancer (BC). (a) Interaction between m6A regulators in BC. Red dots represent erasers, orange dots represent readers, and gray dots represent writers. The line connecting the m6A regulatory factors represents the interaction between them. Pink represents a positive correlation, and blue represents a negative correlation. The size of each circle represents the prognostic effect of each adjustment factor and is scaled by *P* value. Purple indicates a risk factor, and green indicates a protective factor. Using the ConsensusClusterPlus algorithm, BC samples were divided into three m6A modified subclasses, m6Aclusters A, B, and C. (b) Consensus matrix, (c) CDF graph, and (d) relative change of the area under the CDF curve when *k* = 2–9.

**Figure 3:** Related biological pathways and immune landscape characteristics of different m6A modification modes in breast cancer. GSVA enrichment analysis showed the biological pathways in three different m6A modification modes. Heat maps were used to visualize these biological processes. Red represents activated pathways, and blue represents inhibited pathways. (a) m6Acluster A vs. m6Acluster B; (b) m6Acluster A vs. m6Acluster C; (c) m6Acluster B vs. m6Acluster C; (d) CIBERSORT algorithm was used to evaluate the characteristics of immune infiltration between three m6A modification patterns. m6Acluster C showed a better interstitial score, immune score, and ESTIMATE score. (e) Abundance of immune-infiltrating cells in each tumor microenvironment in three different m6A modification patterns in breast cancer (^*∗*^*P* < 0.05, ^*∗∗*^*P* < 0.01, and ^*∗∗∗*^*P* < 0.001).

**Figure 4:** Transcriptome characteristics between different m6A modification patterns in breast cancer. (a) Principal component analysis revealed significant differences in the transcriptome between different m6A modification patterns. (b) Venn diagram showing the differentially expressed genes among the three m6A clusters. GO enrichment analysis was used to annotate m6A-related genes: (c) GO pathway and (d) KEGG pathway.

**Figure 5:** Unsupervised cluster analysis of differentially expressed genes related to prognosis, and patients were divided into three different genomic subtypes (gene clusters A–C): (a) consensus matrix, (b) CDF graph, and (c) relative change in the area under the CDF curve when *k* = 2–9. (d) Principal component analysis showing evident clustering among the three gene clusters. (e) Heat maps showing that these subgroups have different clinicopathological characteristics. (f) Kaplan–Meier was used to analyze the survival curve between different m6A gene clusters. Gene cluster II was associated with better survival outcomes. (g) Expression of m6A regulatory factors in breast cancer in three gene clusters. (h) Abundance of immune-infiltrating cells in three different m6A gene clusters in breast cancer (^*∗*^*P* < 0.05, ^*∗∗*^*P* < 0.01, and ^*∗∗∗*^*P* < 0.001).

**Figure 6:** Construction of m6A gene signature and exploration of its clinical significance. (a) Alluvial diagram showing the changes in m6Aclusters, gene clusters, m6Ascore, and survival status. (b) Correlation between m6Ascore and immune cells based on Spearman analysis. Blue and red indicate negative and positive correlations, respectively. (c) Kruskal–Wallis test was used to compare the difference in the m6Ascore between three different m6A modification patterns. (d) Kruskal–Wallis test was used to compare m6Ascore differences between three different m6A gene clusters. (e) Kaplan–Meier curve was used to analyze the survival of patients in the high- and low-m6Ascore groups. Patients in the low-m6Ascore group showed better survival outcomes. (f) Tumor mutation burden between different m6Ascore groups. (g) m6Ascore and tumor mutation burden (TMB) were negatively correlated (*R* = 0.26, *P* = 8e−16). (h) Kaplan–Meier curve was used to analyze patient survival results between high- and low-TMB groups. (i) Kaplan–Meier curve was used to analyze the survival of patients in the subgroup of m6Ascore and TMB. In both the high- and low-m6Ascore groups, patients in the low-TMB group showed a significant survival advantage. Tumor somatic mutation waterfall chart established from patients with high and low m6Ascores: (j) high-m6Ascore group and (k) low-m6Ascore group. Each upper bar graph shows the TMB, and the number on the right represents the mutation frequency of each gene. The columns represent individual patients.

**Figure 7:** m6Ascore prediction of immunotherapy effects. (a) Relative distribution of TIDE was compared between the high- and low-m6Ascore groups. Treatment effects of CTLA-4 or PD-1 and combined CTLA-4 and PD-1 were evaluated in patients with high and low m6Ascores: (b) CTLA-4 treatment group, (c) PD-1 treatment group, and (d) CTLA-4 and PD-1 combined treatment group. (e) Difference in PD-L1 expression between the high- and low-m6Ascore groups (*P*=0.00018).

## Data Availability

The BC dataset was downloaded from the TCGA database (https://tcga-data.nci.nih.gov/tcga/) and the GEO database (http://www.ncbi.nlm.nih.gov/geo/).
